The article "Analysis of O2O Teaching Assistant Mode of College English in MOOC Environment" was retracted in 2023. Reasons: signs of a paper mill; suspected computer-generated content; unreliable results or conclusions; concerns about the data.

# Analysis of O2O Teaching Assistant Mode of College English in MOOC Environment

**DOI:** 10.1155/2022/8164934

**Published:** 2022-06-29

**Authors:** Yan Zhang

**Affiliations:** Huanghe Jiaotong University, Wuzhi, Jiaozuo 454950, China

## Abstract

In the past, teaching assistants always focused on the physical environment and actions, resulting in a lot of carbon emissions and material waste. This paper discusses the online and offline integration of college English teaching assistance model, which helps inspire the significance of saving energy and reduce carbon emissions in higher education environment. Our country has been putting education informationization in a very important position. In recent years, the demand of college education informatization is more urgent, which calls for the reform of college classroom teaching mode. “O2O teaching mode” is a teaching mode that integrates online and offline teaching, uses computer information network technology, makes use of network media, and relies on online MOOC platform to carry out online network learning and offline face-to-face classroom learning. “O2O teaching mode” has the characteristics of openness, interactivity, individuality, convenience, and generation, which is conducive to changing students' learning mode and teachers' teaching mode, realizing resource sharing, and improving teaching quality. English is a practical course. In the practice of modern English teaching, it is necessary to maintain and develop the advantages of traditional humanistic teaching, and to make efficient use of the media resources and network resources under the condition of modern educational technology, so as to ensure that English learners have active and sufficient practice opportunities. With the popularity of the Internet and the development of MOOC, more and more English learners begin to learn independently online. English online learning platform has become an indispensable tool for independent learning and daily English teaching. Especially when the Internet is connected with the campus network, the role of the network has changed from teaching auxiliary resources to teaching platform, making online learning become a new way of learning, realizing the interaction of English teaching in the network environment.

## 1. Introduction

The development of the times has forced continuous innovation in education, and the advantages of the “Internet plus” teaching model have been fully reflected in the impact of the epidemic [1]. I believe you are no longer unfamiliar with such new words as “opposite classroom,” “Internet +,” “MOOC,” and “O2O.” In order to keep up with the times and the pace of education reform, and to better improve the teaching effect, the author tries to integrate O2O teaching mode into the teaching mode of opposite classroom, in order to achieve the ideal teaching state. Pioneered by Professor Zhang Xuexin, the idea is based on the theories of psychology and educational psychology, in which classes are roughly divided in two, with half of class time allocated to teachers and the other half to students for discussion. At the same time, teachers' teaching time and students' discussion time are separated, so that students can arrange their own learning after class and carry out personalized internalization and absorption. It is worth noting that the discussion in the split mode is in the second class. From the perspective of time schedule, it means that the content taught in the last class is discussed in this class. The purpose of “classroom discussion” is to improve the quality of discussion, and only when students are fully prepared can they discuss actively, have something to say, and enhance their enthusiasm and initiative in learning [2]. The Online to Offline (O2O) teaching model based on Massive Open Online Resources (MOOC) can make students better “prepared” for English teaching and enable the effective implementation of separate classes. In order to deal with the special situation of the epidemic, various teaching platforms poured out during this period, providing students with more excellent teaching courseware, micro video, open class, demonstration class video, and online live broadcast of all kinds of famous teachers' classes. Undoubtedly, this has brought more convenience to education and enriched the learning content of students [3]. The O2O teaching model is a new education model proposed by Qingda learning bar by referring to some experience in the business field and closely connecting with the actual needs of students and parents [4]. The application of this model in auxiliary classroom can make reasonable use of excellent educational resources and improve the effectiveness of learning.

The article "Analysis of O2O Teaching Assistant Mode of College English in MOOC Environment" was retracted in 2023. Reasons: signs of a paper mill; suspected computer-generated content; unreliable results or conclusions; concerns about the data.

Constructivism theory holds that learners do not passively receive external information but actively select and process it. They do not complete the same processing activities under the unified guidance of teachers, but with the assistance of teachers and others, they construct their meanings to the real world through unique information processing activities [5]. According to the Basic Requirements of English Teaching for Higher Vocational Education by the Ministry of Education, vigorously introducing and applying all kinds of advanced teaching methods can cultivate students' interest and enthusiasm in English learning, so as to strengthen students' ability to consciously learn English. O2O MOOC points the classroom environment, and the theoretical basis of the auxiliary teaching mode mainly follows the built socialism theory, by adopting the combination of online teaching way to a full range of English learning and, at the same time, giving full play to the guidance of teachers in the classroom, guiding and helping learners fully participate in the whole learning process and the initiative to build knowledge learning [6].

MOOC is a large-scale web development course, which is characterized by diversification, wide audience, and easy operation. The English MOOC teaching system can check the teaching tasks and analyze the overall teaching effect by virtue of online technology and background data statistical analysis. Under the MOOC environment, the O2O teaching assistant mode of English teaching in higher vocational colleges makes use of MOOC network resources to enable students to further consolidate and learn the content taught by teachers and then internalize it into their own, so as to be well prepared to participate in the discussion. Therefore, in a sense, the divided class is essentially to introduce an internalized link of psychology between teaching and discussion and realize the unity of opposites between “teaching method” and “learning method” through the organic integration of teaching and discussion [7]. O2O MOOC environment auxiliary teaching mode in effective internalization of this link can be twice the result with half the effort, and it can integrate students' learning knowledge of English, and refining and summarizing, with corresponding strategies, help students' learning ability play itself to the best condition and, at the same time, stimulate students' learning enthusiasm and set up the higher consciousness of autonomous learning.

Firstly, under the guidance of constructivism and based on MOOC, this paper builds an O2O teaching platform for non-English majors in higher vocational colleges, focusing on the construction of learning database.

Secondly, combined with the O2O teaching platform and flipped classroom model, the O2O teaching model of Vocational English is constructed, and the feasibility and effectiveness of the model are verified. The platform from the angle of the users is divided into learners, teachers, and teacher three roles, giving priority to the learning and learners' online autonomous learning function, and according to the function of the system, thr partition could be divided into independent learning platform system, resource management system, teaching management system, evaluation feedback system, certification system, etc. All the self-learning content in the platform is embodied in the form of tasks to improve the enthusiasm of learners for self-learning.

The article "Analysis of O2O Teaching Assistant Mode of College English in MOOC Environment" was retracted in 2023. Reasons: signs of a paper mill; suspected computer-generated content; unreliable results or conclusions; concerns about the data.

Finally, this paper applies O2O teaching model to conduct teaching experiment research. This study took students from two classes of foreign-related nursing major in a vocational and technical college in Fujian as the experimental objects and compared the teaching effects of O2O teaching mode based on MOOC and 3P teaching mode in vocational English through experiments. The experimental results show that there is a significant difference between the scores of the experimental class and the control class, which proves that the O2O teaching mode of higher vocational English has certain effectiveness and feasibility. If the mode is properly used in English teaching, it will help strengthen the enthusiasm of higher vocational students to learn and improve their practical English application ability.

On the one hand, the research of this paper enriches the theory of English teaching and has theoretical significance. On the other hand, it can also provide reference for practical teaching and has practical significance.

## 2. State of the Art

In the past two decades, the cognitive learning theory that advocates students as the subject of information processing has replaced the behaviorist learning theory that regards students as the object of knowledge indoctrination. In recent years, psychologists continue to carry out in-depth research on the cognitive law of human learning process, which makes constructivism learning theory, an important branch of cognitive learning theory, become gradually popular in the educational circle. “Although it is impossible to complete the establishment of constructivist theoretical system in the short term, its core ideas and basic principles have been established, which can provide practical guidance for the teaching design of constructivist learning environment based on Internet and multimedia technology.” Its guiding principles are as follows:

Being student-centered is not only the basic idea and starting point of online autonomous learning, but also the core content of online autonomous learning teaching theory and learning theory [8]. “Initiative, externalization of knowledge, and self-feedback are the three basic elements to achieve student-centered development.”

The learning context must be conducive to the meaning construction of the essence of the learning content (that is, the understanding of the learning content) and can complete the meaning construction of new knowledge through “assimilation” and “adaptation.” Therefore, teaching design should not only analyze teaching objectives, but also take situation creation as one of the main contents of teaching design, which is beneficial to learners to construct meaning. However, in the traditional classroom mode, it will be difficult for learners to construct the meaning of knowledge because learners cannot be provided with vivid and practical situations.

The article "Analysis of O2O Teaching Assistant Mode of College English in MOOC Environment" was retracted in 2023. Reasons: signs of a paper mill; suspected computer-generated content; unreliable results or conclusions; concerns about the data.

“Collaborative learning, whether between teachers and students or between students and students, plays an important role in the collection and analysis of learning materials, the proposal and verification of teaching hypotheses, the evaluation of learning outcomes, and the ultimate construction of meaning” [9].

Teaching design under the guidance of constructivism is not the design of teaching environment, but the design of learning environment. The interaction between learner and learning environment plays a key role in the construction of knowledge meaning. Learning environment refers to the place where learners study independently and explore freely. In this environment, learners can use various information resources and learning tools (such as books, text materials, audio-visual materials, network information, CAI, and multimedia courseware) to achieve their learning goals. Learning should be supported and facilitated, not strictly controlled. The learning environment is a place that supports and promotes autonomous learning.

“In order to promote learners to actively explore and achieve meaning construction, learners must be provided with various types of information resources, including various teaching materials and teaching media; however, these materials and media are not used to support teachers' lecture and demonstration, but to assist learners' autonomous learning and collaborative exploration.” In the process of learners' active exploration, teachers are in urgent need to provide guidance and help on the acquisition methods, acquisition approaches, and effective processing and utilization of all kinds of information resources [10].

Constructivism theory holds that “the meaning to be constructed refers to the law and nature of things and the internal connection between things.” The learning process of helping learners to achieve meaning construction is to help learners to have a deep understanding of the laws, nature, and internal relationships of things contained in the current learning content [11]. In constructivism learning environment, learners are emphasized as cognitive subjects and active constructors of meaning, so the realization of meaning construction of knowledge by learners is the ultimate goal of the whole learning process, and the whole teaching design must be subordinate to the center of “meaning construction.”

The article "Analysis of O2O Teaching Assistant Mode of College English in MOOC Environment" was retracted in 2023. Reasons: signs of a paper mill; suspected computer-generated content; unreliable results or conclusions; concerns about the data.

Whether we can get rid of the shackles of traditional teaching mode is the key point of deepening teaching reform at home and abroad [12]. This traditional teacher-led teaching mode suppresses the initiative of students as cognitive subjects and is difficult to undertake the responsibility of cultivating high-quality talents with practical ability and innovative spirit. In order to achieve the goal of teaching reform, experts and scholars at home and abroad have carried out a great deal of in-depth exploration and research from both theoretical and practical levels over the years, and constructivism theory is one of the important achievements. With the wide application of Internet and multimedia technology in the field of education, the influence of constructivism theory is expanding day by day all over the world. However, it is still worth thinking how to apply the theory into the demonstration teaching and how to use the demonstration to prove its feasibility, which is discussed in this paper.

## 3. Methodology

### 3.1. Research on Online Autonomous Learning System

There have been a lot of in-depth studies on online autonomous learning at home and abroad. Tables 1 and 2 are statistics of research papers and websites or web pages related to online autonomous learning found by keywords in the three global search engines and CNKI respectively.

Since the 1950s, many disadvantages of the traditional education model have led to the stagnation of the study of educational methods. Some educational experts have gradually shifted their research focus from the study of educational objectives, educational methods, and educational content to the study of learning methods for learners, resulting in many learning theories [13]. Since the 1970s, many schools of psychology have studied autonomous learning from different perspectives, and learners have been attached great importance. The theory and practice of autonomous learning have become a hot issue in educational research and educational psychology. Psychologists led by Zimmerman B. J. put forward a set of influential autonomous learning theory in the 1990s. Zimmerman B. J. explained the essence of autonomous learning from six aspects of learning motivation, method, behavior, time, social environment, and material environment. In terms of educational practice, scholars have also carried out practical research on teaching modes that promote students' autonomous learning ability, for example, “Manning's cognitive self-guidance model, Johnson's cooperative learning model, Machenbaum's speech self-guidance training program, and the educational reform of Okawa Gakuen in Japan under the guidance of Kohara's Whole Person Education Theory.”

The article "Analysis of O2O Teaching Assistant Mode of College English in MOOC Environment" was retracted in 2023. Reasons: signs of a paper mill; suspected computer-generated content; unreliable results or conclusions; concerns about the data.

At the same time, the rapid development of online education in foreign countries also drives the research on online autonomous learning system and the development of online autonomous learning. The main performance is as follows:

Lindenlaub John in the article “A Hybrid Lecture/Self-study System for Large Engineering Classes” mainly expounds the study of the learning environment in the autonomous learning System and also studies the autonomous learning methods and characteristics of autonomous learning. By comparing the traditional course arrangement and materials with those in the independent learning system, Lindenlaub John pointed out that the independent learning environment has a certain influence on the independent learning method, and the learning method in the independent learning system is more flexible than the traditional learning method [14].

Wilder in an Individual self-study System in A Numerical Mathematics Course Based on Educational “Software” describes an independent learning system designed for sophomore engineering courses. The author analyzes the impact of the independent learning system on learners' learning from three aspects: the development of independent learning materials, the change of evaluation methods, and the development of learning tools. Due to the influence of these three aspects, learners' online independent learning is more planned and regular compared with offline independent learning.

### 3.2. O2O Teaching Model Introduction

There are various versions of the connotation of “O2O teaching mode.” Based on the views of other scholars, the author summarizes the connotation of “O2O teaching mode” as follows: O2O teaching mode mainly refers to the use of computer information network technology, with the help of network media. Relying on online MOOC platforms (such as Good University Online and UOOC Alliance), the teaching mode is highly combined with online network learning and offline face-to-face classroom learning. This hybrid teaching model allows students to achieve personalized learning goals through online learning while attending in-person on-campus classes. The schematic diagram is as follows in Figure 1:

#### 3.2.1. Characteristics of Learning under O2O Teaching Mode

A typical O2O teaching mode is shown in Figure 2. The characteristics of this mode of learning are as follows: online MOOCs videos explain basic knowledge of the course and use network media to carry out video, voice, forum Q&A, and other forms of interaction. Passing the pass requires students to complete online coursework, exams, etc. Offline, teachers of each course group will carry out special teaching based on textbooks and students' majors, guide students to carry out small-class discussions after class online, and organize students to participate in relevant social practice activities.

The article "Analysis of O2O Teaching Assistant Mode of College English in MOOC Environment" was retracted in 2023. Reasons: signs of a paper mill; suspected computer-generated content; unreliable results or conclusions; concerns about the data.

#### 3.2.2. Characteristics of Assessment under O2O Teaching Mode

Figure 3 shows the activity flow of a typical O2O teaching model. Online examination is mainly composed of teachers and teaching assistants to complete, but the characteristics of “peer mutual links, namely, between learners and learners, can also be mutual comparison, all students who complete online learning tasks, such as watching video, complete online assignments, and all kinds of test, participate in the BBS and mutual teaching, etc., and through online and offline test with qualified score, and confirmed by the curriculum group, students who meet the credit requirements of the school will be recognized as course credits by the school according to its regulations.

Hybrid learning mode is the general trend of the future development of higher education in China, and it is an important support for teaching and learning to improve students' personal ability. It is not just a simple use of advanced network technology as a teaching aid tool, but also integrates itself into the main part of teaching. The assessment method of O2O teaching mode is that those whose total score of online evaluation system evaluation and peer mutual evaluation exceeds the passing score can be granted half of the credits of the course, and those whose total score of offline final assessment and practice report exceeds the passing score can be granted the other half of the credits of the course. Full credits will be awarded to students who have completed both online and offline tests [15]. Based on this, the two constitute an organic and complete teaching process. The Christensen Institute cited graded change and blended learning as examples. A key factor in most definitions of blended learning is that students must learn to control their time and develop their ability to choose a path or rate of learning. With the advent of the era of the Internet + mobile Internet, mobile client education APP classes will give the future of the application of the hybrid education mode to add more support to students' fragmentation and online learning time and support their personalized learning habits, and the system will default to support learners learning rhythm to remind the time to study at ordinary times, or the complete practice work. At the same time, this powerful function is also applicable to teachers.

### 3.3. Current Situation and Analysis of MOOC Research

#### 3.3.1. Foreign Research and Application of MOOC

MOOC originated in the United States in the late 1990s. In 2008, the Canadian academics Bryan Alexander and Dave Cormier jointly coined the term “MOOC.” This massive MOOCs took higher education by storm in the fall of 2011, heralded as “the biggest innovation in education since the invention of printing” and heralded the “future of education.” The New York Times described 2012 as “the first year of MOOCs.” As of May 2013, there were about 450 MOOCs around the world, and the number is still growing. The leading MOOCs providers in the US are Coursera, edX, and Udacity. About 20 schools in the UK have started offering free online courses using the Future Learn platform. MOOC providers have also sprung up in other countries, such as Iversity in Germany, School in Japan, Veduca in Brazil, and more. MOOCs in the United States have partnered with universities in Australia, China, Switzerland, and other countries. The interactive relationship between online activities and offline activities is shown in Figure 4.

The article "Analysis of O2O Teaching Assistant Mode of College English in MOOC Environment" was retracted in 2023. Reasons: signs of a paper mill; suspected computer-generated content; unreliable results or conclusions; concerns about the data.

#### 3.3.2. Domestic Research and Exploration of MOOC

At present, the construction of MOOC in China is in the initial and exploratory stage [16]. The year 2013 is known as “the first year of Chinese MOOC.” MOOC development in China and the world is almost synchronous. The new era of education represented by MOOC has come. EdX, one of the so-called “MOOC troika,” announced the addition of online courses at 15 universities, including six Asian universities including Peking University and Tsinghua University. In July 2013, Fudan University and Shanghai Jiaotong University signed contracts with Coursera. In a short period of time, the frequent interaction between Chinese famous universities and MOOC companies proves that MOOC, a new education model, has brought a huge impact on China's higher education. With the cooperation, MOOC platforms in the United States will offer courses from Chinese universities for the first time. According to the agreement, Coursera must subtitle a course within seven working days if 10,000 people have signed up for it. Fudan University, Shanghai Jiaotong University, and other universities will offer online courses to the world, building the world's largest online course network together with Harvard, MIT, and Stanford. About 130,000 Chinese users registered on Coursera in 2013, ranking ninth in the world, according to the company. In 2014, the figure was 650,000, a far larger increase than in any other country.

Meanwhile, Chinese universities are building their own MOOC platforms. Led by Shanghai Jiaotong University, C9 universities such as Peking University, Tsinghua University, Zhejiang University, Fudan University, NTU, Xi'an Jiaotong University, Harbin Institute of Technology, and China University of Science and Technology, as well as Tongji University, Dalian University of Technology, and Dalian University of Technology, jointly built the “China MOOC” [17]. The above universities will strengthen cooperation in the curriculum standards and construction of “open online courses,” the construction of sharing platform and sharing mechanism, and jointly explore the training mode of cross-school joint minor based on MOOC. The curriculum characteristics of the constructed MOOC have the characteristics shown in Figure 5.

The article "Analysis of O2O Teaching Assistant Mode of College English in MOOC Environment" was retracted in 2023. Reasons: signs of a paper mill; suspected computer-generated content; unreliable results or conclusions; concerns about the data.

### 3.4. Differences with Traditional 3P English Teaching Model

“The traditional 3P English Teaching model is a CL-communicative Language Teaching developed in the 1970s on the basis of behavioral psychology and structuralist linguistics”; the so-called 3P refers to the three stages of language teaching: Presentation, Practice, and Production. In the process of English teaching, the teacher first presents the language knowledge through teaching and then lets the students master the language knowledge in the practice. Finally, under the controlled or semicontrolled state, let the students carry on the hypothesis communication and realize the language output, so as to complete the teaching process.

The pattern of students in the class teaching target required to master the English language form, the student by the English teacher in a language independent project explained and classroom practice, can in one pace reach the designated position to master the content of classroom teaching and use, with teaching and promoted learning, thinking that as long as the teacher explained, students could master, and in fact, it is hard to achieve this goal. Its classroom teaching form focuses on language input, emphasizing the mechanical practice and accumulation of language knowledge. This kind of simple and crude knowledge indoctrination plus monotonous and boring language practice is easy to have a negative impact on students' learning interest and enthusiasm; in teaching evaluation, teachers generally adopt summative evaluation (examination and test, etc.), usually focusing only on learning results.

The advantages of this mode are as follows: first of all, it ensures teachers' dominance, facilitates teachers' classroom organization and management, and improves the effectiveness of classroom teaching. Secondly, it emphasizes the controllability of teaching, which can effectively guarantee the systematic teaching of language structure and form. Finally, paying attention to the participation of students, students' practice is carefully designed by teachers, which is conducive to achieve the best teaching effect.

The article "Analysis of O2O Teaching Assistant Mode of College English in MOOC Environment" was retracted in 2023. Reasons: signs of a paper mill; suspected computer-generated content; unreliable results or conclusions; concerns about the data.

However, this mode is also accompanied by self-evident defects: first, the 3P mode is a teaching mode of one-way knowledge transfer centered on “teaching before learning,” which ignores the real needs and learning status of students [18]. Second, the 3P mode is limited by time and space, so it is difficult to set personalized teacher-student interaction and teaching schedule. Thirdly, 3P mode emphasizes English language form rather than language content, which leads to imbalance between the two. Fourthly, due to the emphasis on language forms, the compilation of teaching syllabus is mainly based on grammar, which is difficult to take into account the rules of grammar acquisition of second language learners and cannot internalize the development system of interlanguage grammar of second language learners.

## 4. Result Analysis and Discussion

This study will compare and analyze the difference in teaching effects caused by 3P teaching mode and MOOC-based O2O teaching mode of vocational English through experiments, so as to explore the feasibility of MOOC-based O2O teaching mode of vocational English.

### 4.1. The Experimental Process

For data availability and scientific reliability reasons, the samples of this experiment came from two classes with similar average scores in foreign nursing major of a vocational and technical college in Fujian and were randomly divided into experimental class and control group [19]. The experimental class (52 students) adopts the VOCATIONAL English O2O teaching mode, while the control class (51 students) adopts the traditional 3P teaching mode. The two classes are completely the same in teaching materials, teachers, class hours, and other aspects, but the only difference is the adoption of different teaching modes. Using this sample, we can better compare the learning gap between classes under different teaching modes.

In the teaching process, the author adopts the O2O teaching mode of Higher vocational English for the experimental class, focusing on the use of MOOC video platform resources to guide students to conduct online autonomous learning, while the control class continues the traditional 3P teaching mode, focusing on classroom teaching. As shown in Table 3, the author took New Horizons English Course Unit 4Science and Technology as the classroom Teaching example.

### 4.2. Analysis of Experimental Results

The test paper is of grade B of the National College English Application Ability Test, as seen in Tables 4–9. The result is used as the pretest result. Then, the independent sample *T* test was used for statistical analysis of the pretest scores of the experimental class and the control class, and there was no significant difference in the English pretest scores of the two groups (*P*=0.210 > 0.05). The test is to compare the differences between the two groups of data, whether there is statistical significance; the premise of *t*-test is that the two groups of data are from normally distributed groups, and the variance of the data is uniform, which satisfies the independence. Independent sample *T* test (there is no correlation between experimental treatment groups, that is, independent samples) is used to test the difference of data obtained by two groups of unrelated samples. Therefore, before the teaching experiment, the starting point of the experimental class and the control class was the same, and there was no significant difference in the English level [20].

The article "Analysis of O2O Teaching Assistant Mode of College English in MOOC Environment" was retracted in 2023. Reasons: signs of a paper mill; suspected computer-generated content; unreliable results or conclusions; concerns about the data.

At the same time, the author also used paired sample *T* test to make a comparative analysis of the pre- and posttest scores of the experimental class and the control class, respectively. *T* test results of paired design samples before and after test results of experimental classes were *T* = −8.764, DF = 51, *P* value of bilateral test (Sig.) = 0.000 < 0.005, indicating that there were significant differences in the test results before and after test results of experimental classes [21]. The *t*-test result of paired design sample of the control class's pre- and posttest scores is *T* = −1.646, DF = 50, and *P* value (Sig.) = 0.106 > 0.005, indicating that the pre- and posttest scores of the control class are improved, but there is no significant difference. The above experimental results show that, compared with the traditional English 3P teaching mode, higher vocational English O2O teaching model can improve students' English scores on the whole.

In this experiment, the national standardized examination papers were used for both pretest and posttest, and the examination process was supervised by camera. In order to ensure the reliability and validity of the test results, the English teaching and Research Section of the college arranged the flow marking.

The statistical results show that the pretest and posttest scores of both the experimental class and the control class are normally distributed, while the posttest scores of the experimental class are significantly higher than those of the control class. The difference between the two is significant, indicating that the O2O teaching mode of English in vocational colleges is indeed conducive to improving the teaching effect [22]. The experimental results show that the O2O teaching mode of Higher vocational English has a significant positive correlation with the learning effect of higher vocational students, which has certain effectiveness and feasibility. Through empirical comparison, we can see the superiority of the English teaching model adopted in this paper, which provides empirical evidence for the demonstration of this paper.

The article "Analysis of O2O Teaching Assistant Mode of College English in MOOC Environment" was retracted in 2023. Reasons: signs of a paper mill; suspected computer-generated content; unreliable results or conclusions; concerns about the data.

Students' satisfaction with online teaching is shown in Figure 6:

## 5. Conclusion

In order to improve the quality and effect of higher vocational English teaching and better design of higher vocational English courses, this paper constructed a new O2O higher vocational English teaching model, focusing on the construction of O2O teaching platform based on contains, and improving the traditional 3 P English teaching model. And this article carries on the empirical test to the two teaching modes. In this paper, the experimental samples were selected from two classes of foreign-related nursing major in a vocational and technical college of Fujian, which were randomly divided into experimental class and control group. The experimental class (52 students) adopts the vocational English O2O teaching mode, while the control class (51 students) adopts the traditional 3P teaching mode. The two classes are completely the same in teaching materials, teachers, class hours, and other aspects, but the only difference is the adoption of different teaching modes.

In the teaching process, the author adopts the O2O teaching mode of higher vocational English for the experimental class, focusing on the use of MOOC video platform resources to guide students to conduct online autonomous learning, while the control class continues the traditional 3P teaching mode, focusing on classroom teaching. Through empirical analysis, this paper finds that using MOOC video platform resources to guide students to conduct online autonomous learning has better learning efficiency.

On the one hand, through the analysis and summary of a large number of domestic and foreign literature, and a questionnaire survey of English autonomous learning of vocational college students, so as to determine the construction scheme of O2O teaching platform resource management system in vocational College English, based on the theory of constructivism, it integrates the advantages of MOOCs and flipped teaching and designs an O2O teaching model suitable for vocational college students, which is compatible with online and offline teaching methods.

On the other hand, this paper conducts an experimental study on the MOOC-based O2O teaching mode of higher vocational English [23]. This study takes two classes of nursing major in a vocational and technical college in Fujian as the experimental objects, compares and analyzes the differences between the two teaching modes through experiments, and makes statistical analysis on the experimental results with SPSS19.0. This paper proves that the O2O teaching mode of higher vocational English has certain effectiveness and feasibility, and the rational use of this mode in teaching can help enhance students' learning initiative and improve their English practical application ability.

The article "Analysis of O2O Teaching Assistant Mode of College English in MOOC Environment" was retracted in 2023. Reasons: signs of a paper mill; suspected computer-generated content; unreliable results or conclusions; concerns about the data.

The result of this teaching reform means that higher vocational English teaching has been promoted to a new level, especially the O2O teaching platform of higher vocational English based on MOOC has provided strong support for higher vocational students to improve their autonomous learning ability.

It is often said that “there is a method in teaching, but there is no fixed method in teaching. It is important to get the method and innovate the method.” All kinds of new theories and methods of English teaching emerge endlessly, but any kind of teaching model inevitably has some shortcomings and defects, and so does the O2O teaching model of English in vocational colleges. Although online autonomous learning can well achieve relevant educational goals, it cannot completely replace traditional 3P classroom teaching, let alone school education. Therefore, the two teaching modes can permeate and complement each other, combining online autonomous learning with offline classroom teaching. Only by adopting the corresponding teaching mode according to the actual situation of teaching can we promote the transformation of English language knowledge into English language skills and the formation and development of learners' comprehensive English language ability. At the same time, from the comparative research experiment of the two teaching modes, we can find that higher vocational English O2O teaching mode has certain advantages and advanced, but how to deeply explore the deep potential and application value of this teaching mode and really play the role of HIGHER vocational English O2O teaching platform and online autonomous learning in English learning, so as to provide a certain theoretical and practical basis for the future development of Vocational English teaching, is still a problem to be further studied and discussed.

To sum up, in the application of English classroom teaching method, we can find an appropriate meeting point between form and content, so that we can utilize the O2O teaching mode of English in vocational colleges and organically combine the traditional 3P teaching mode and online autonomous learning mode in the MOOC environment. The English teaching experiment we try under the guidance of constructivism theory has a certain theoretical basis and practical significance, and the teaching plan designed under the guidance of this theory can indeed promote the development of English classroom teaching method and achieve the purpose of enhancing the effect of classroom teaching.

The article "Analysis of O2O Teaching Assistant Mode of College English in MOOC Environment" was retracted in 2023. Reasons: signs of a paper mill; suspected computer-generated content; unreliable results or conclusions; concerns about the data.

## Figures and Tables

**Figure 1:** Two cycle modes of MOOC.

**Figure 2:** Higher vocational English O2O teaching platform.

**Figure 3:** O2O teaching mode of higher vocational English.

**Figure 4:** Online and offline teaching.

**Figure 5:** MOOC curriculum characteristics.

**Figure 6:** Students' satisfaction with online learning.

**Table 1:** The number of relevant web pages searched by the three major search engines.

Search engine	Keyword		
	Online self-directed learning	e-learning	MOOC
Google	1,110,000	187,000,000	9,210,000
Yahoo	1,120,000	49,990,000	1,460,000
Baidu	7,700,000	7,440,000	967,000

**Table 2:** The number of related papers searched by CNKI.

Dissertation database	Keyword		
	Online self-directed learning	e-learning	MOOC
Full-text database of Chinese periodicals	40,947	9,771	1,549
The full text of China's outstanding doctoral and master's degree thesis	10,268	3,387	82

**Table 3:** Examples of classroom teaching.

	Experimental class	Comparative class
Teaching goal	Vocabulary. grade A3/B22/superclass 6grammar: adjoint adverbial (adjoint adverbial) text: understand and repeat. Listening and speaking: understanding and expressing. Vocabulary. grade A3/B22/superclass 6grammar: adjoint adverbial (adjoint adverbial) text: understand and repeat. Listening and speaking: understanding and expressing	Vocabulary. grade A3/B22/superclass 6grammar: adjoint adverbial (adjoint adverbial) text: understand and repeat. Listening and speaking: understanding and expressing. Vocabulary. grade A3/B22/superclass 6grammar: adjoint adverbial (adjoint adverbial) text: understand and repeat. Listening and speaking: understanding and expressing
Teaching mode	English O2O teaching model in higher vocational education	3P teaching mode
Curriculum evaluation system	Formative evaluation (result of debate) + (final exam) price (platform unit clearance test)	Final evaluation (unit small test + midterm exam)
Instructor	The author (supplementary 1 class hour) foreign teacher (classroom discussion 1 class hour)	The author (4 hours in the text) the foreign teacher (2 hours of listening and speaking training)
Teaching process	I preclass autonomous learning (2 hours): students learn autonomously on the teaching platform and complete the online communication and feedback of the platform test.	I Introduction + text explanation (2 hours) II grammar explanation and practice (2 hours) III listening and speaking training (2 hours)
	*II classroom learning (2 hours):*	

Oral classroom content	II after class autonomous learning (2 hours): students complete unit test platform to expand learning online communication and feedback on the teaching platform. Organize students to “is the development of modern science and technology bringing happiness or misfortune to mankind?” group debate for the debate (1 class hour of discussion)	Organize students to “is the development of modern science and technology bringing happiness or misfortune to mankind?” group debate for the debate (1 class hour in oral English)

The article "Analysis of O2O Teaching Assistant Mode of College English in MOOC Environment" was retracted in 2023. Reasons: signs of a paper mill; suspected computer-generated content; unreliable results or conclusions; concerns about the data.

**Table 4:** Comparison of pretest results.

Group	Number of people	Mean	Standard deviation	The standard error of the mean
Experimental class	52	78.0192	8.011	1.11093
Control class	51	75.8627	9.03165	1.30249

**Table 5:** Independent sample *T* test.

	*F*	Sig.	*T*	df	Sif (bilateral)	Mean difference	Standard error value	95% confidence interval for difference	
								Lower bound	Upper bound
Assume that the variances are equal	3.06	0.083	1.262	101	0.21	2.15649	1.70942	−1.23455	5.54752
Assume that the variances are not equal			1.26	98.238	0.211	2.15649	1.71191	−1.24064	5.55362

**Table 6:** Comparison of posttest results.

Group	Number of people	Mean	Standard deviation	The standard error of the mean
Experimental class	52	84.0385	6.1356	0.85085
Control class	51	78.5686	7.85431	1.09982

**Table 7:** Independent sample *T* test.

	*F*	Sig.	*t*	df	Sif (bilateral)	Mean difference	Standard error value	95% confidence interval for difference	
								Lower bound	Upper bound
Assume that the variances are equal	3.15	0.079	3.943	101	0	5.46983	1.38723	2.71794	8.22173
Assume that the variances are not equal			3.934	94.555	0	5.46983	1.39053	2.70912	8.23055

**Table 8:** Comparison of performance before and after.

		Mean	Number of people	Standard deviation	The standard error of the mean
Control 1	Experimental preclass testing	78.0192	52	8.011	1.11093
	Experimental class posttesting	84.0385	52	6.1356	0.85085
Control 2	Control class pretesting	75.8627	51	9.30165	1.30249
	Control postclass testing	78.5686	51	7.85431	1.09982

**Table 9:** Paired sample *T* test.

		The ingredients are different					*t*	Sif (bilateral)
		Mean	Standard deviation	The standard error of the mean	95% confidence interval for difference			
					Lower bound	Upper bound		
Control 1	EC1-EC2	−6.01923	4.95268	0.68781	−7.39807	−4.6404	−8.764	0
Control 2	EC1-EC2	−2.70588	11.74273	1.64431	−6.00858	0.59681	−1.646	0.106

## Data Availability

The labeled data set used to support the findings of this study is available from the author upon request.

## References

[1] Zheng J., Huang L., Li S., Lajoie S. P., Chen Y., Silver C. E. H. (2021). Self-regulation and emotion matter: a case study of instructor interactions with a learning analytics dashboard. *Computers & Education*.

The article "Analysis of O2O Teaching Assistant Mode of College English in MOOC Environment" was retracted in 2023. Reasons: signs of a paper mill; suspected computer-generated content; unreliable results or conclusions; concerns about the data.

[2] Kochan J. (2020). Subjectivity and emotion in scientific research. *Studies in History and Philosophy of Science*.

[3] Vicky T. L., Huettig F. (2020). When prediction is fulfilled: insight from emotion processing. *Journal of Neuropsychology*.

[4] Gennady G., Knyazev (2020). Motivation, emotion, and their inhibitory control mirrored in brain oscillations. *Neuroscience and Biobehavioral Reviews*.

[5] Xu A., Jennifer E. S., Yang X. (2021). Evolution of emotion semantics. *Cognition*.

[6] Gong Y., Rina S. (2021). Autonomous learning of foreign language based on facial emotion recognition and cloud computing. *Journal of Intelligent and Fuzzy Systems*.

[7] Kopczyk A. B. (2020). Verbs of emotion with se in Slovene: between middle and reflexive semantics. A cognitive analysis. *Cognitive Studies*.

[8] Hosseini A. S. (2017). Sentence-level emotion mining based on combination of adaptive meta-level features and sentence syntactic features. *Engineering Applications of Artificial Intelligence*.

[9] Li H. (2021). Emotions, English language teaching: exploring teachers’ emotion labor. *Journal of Educational Review*.

[10] Marian V., Kaushanskaya M. (2020). Self-construal and emotion in bicultural bilinguals. *Journal of Memory and Language*.

[11] Bloom R. L., Borod J. C., Obler L. K., Koff E. (1990). A preliminary characterization of lexical emotional expression in right and left brain-damaged patients. *International Journal of Neuroscience*.

[12] Kim E. (2022). Prepositions with and about and schematic conceptualisation of emotion causality. *English Studies*.

[13] Morris K. (2020). Fear becomes first emotion to yield to molecular neuroscience. *The Lancet Neurology*.

[14] Michael E. H. (1988). Metamotivation, emotion, and dominance: review of reversal theory: applications and developments. *New Ideas in Psychology*.

[15] Ahmed A., Morgan B (2021). Postmemory and multilingual identities in English language teaching: a duoethnography. *Language Learning Journal*.

[16] Yang S., Shu D., Hongbiao Y. (2021). “Frustration drives me to grow:” unraveling EFL teachers’ emotional trajectory interacting with identity development. *Teaching and Teacher Education*.

[17] Thorley D. (2019). Towards a history of emotion, 1562–1660. *The Seventeenth Century*.

[18] O’Toole Mia S., Emma E., Mai B. M. (2021). Is negative emotion differentiation associated with emotion regulation choice? investigations at the person and day level. *Frontiers in Psychology*.

[19] Qi L., Wang S. (2019). Translation and emotion: a psychological perspective. *Jazz Perspectives*.

[20] Chris B. (1986). *An Attributional Theory of Motivation and Emotion: B. Weiner*.

The article "Analysis of O2O Teaching Assistant Mode of College English in MOOC Environment" was retracted in 2023. Reasons: signs of a paper mill; suspected computer-generated content; unreliable results or conclusions; concerns about the data.

[21] Spada M. M., Nikčević A. V., Moneta G. B., Wells A. (2007). Metacognition as a mediator of the relationship between emotion and smoking dependence. *Addictive Behaviors*.

[22] Acerbi A., Lampos V., Garnett P., Bentley R. A. (2013). The expression of emotions in 20th century books. *PLoS One*.

[23] Hanzhou P. (2019). Individuating emotional clarity in multicultural classrooms of higher education: a transnational study on nonverbal dynamics of enculturation and acculturation. *Cogent Education*.

